# Genetic Engineering of Filamentous Fungi for Efficient Protein Expression and Secretion

**DOI:** 10.3389/fbioe.2020.00293

**Published:** 2020-04-08

**Authors:** Qin Wang, Chao Zhong, Han Xiao

**Affiliations:** ^1^State Key Laboratory of Microbial Metabolism, Joint International Research Laboratory of Metabolic & Developmental Sciences, and Laboratory of Molecular Biochemical Engineering, School of Life Sciences and Biotechnology, Shanghai Jiao Tong University, Shanghai, China; ^2^Materials and Physical Biology Division, School of Physical Science and Technology, ShanghaiTech University, Shanghai, China; ^3^Materials Synthetic Biology Center, Shenzhen Institute of Synthetic Biology, Shenzhen Institutes of Advanced Technology, Chinese Academy of Sciences, Shenzhen, China

**Keywords:** filamentous fungi, genetic engineering, protein secretion, expression, genome engineering

## Abstract

Filamentous fungi are considered as unique cell factories for protein production due to the high efficiency of protein secretion and superior capability of post-translational modifications. In this review, we firstly introduce the secretory pathway in filamentous fungi. We next summarize the current state-of-the-art works regarding how various genetic engineering strategies are applied for enhancing protein expression and secretion in filamentous fungi. Finally, in a future perspective, we discuss the great potential of genome engineering for further improving protein expression and secretion in filamentous fungi.

## Introduction

Protein production has a broad application in life sciences, biotechnology, medicine and material sciences. Filamentous fungi are powerful and efficient cell factories for protein production at the industrial scale, and over half of the commercially available proteins were produced by filamentous fungi^1^. Many species of filamentous fungi are generally regarded as safe (GRAS), and exhibit superior protein secretory capability. For example, 25–30 g/L of glucoamylase was obtained from fermentation medium of *Aspergillus niger*, while *Trichoderma reesei* was able to secret 100 g/L of cellulose (Ward, 2012). Compared to prokaryotes, filamentous fungi own the mature systems for post-translational processing (e.g., glycosylation, protease cleavage, and disulfide bond formation) (Karnaukhova et al., 2007), which are indispensable for protein function and activity. Although yeasts are able to perform post-translational modification, they tend to produce proteins in the form of high mannose-type glycosylation. In contrast, filamentous fungi have less extensive hyper-mannosylation of glycoproteins, which could be directly converted to mammalian type of glycoproteins with pharmaceutical potential (Punt et al., 2002; Deshpande et al., 2008). In addition, due to the metabolic diversity, filamentous fungi can efficiently utilize many types of monosaccharides including xylose, arabinose, and galactose, while yeasts can only metabolize glucose and mannose (Cavka and Jönsson, 2014).

To further improve the production of various proteins by filamentous fungi, traditional strategies including optimization of fermentation process and obtaining beneficial mutants via random mutagenesis, were widely adopted in the past. Here, rather than providing a comprehensive view of achieving efficient protein production, we focus on summarizing the strategies based on genetic engineering of this particular cell factory to enhance protein expression and secretion. We also provide new ideas in terms of cell factory engineering.

## Protein Secretion Pathway in Filamentous Fungi

Protein secretion pathway in filamentous fungi involves three major steps including: polypeptide transfer from ribosome to endoplasmic reticulum (ER), protein folding and modification in ER, transportation of the folded protein vesicles to the Golgi apparatus and extracellular environment (Figure 1). In the first step, the co- or post-translational transport pathway is responsible for the polypeptide transfer from the ribosome to ER. In the co-translational transport pathway, the signal peptide recognition particle (SRP) first binds to the signal peptide sequence to block translation (Halic et al., 2006). Then, SRP directs the ribosome-mRNA-nascent peptide complex to target the ER membrane and binds to the SRP receptor. Subsequently, SRP is released from the complex, translation resumes, and the nascent polypeptide enters ER lumen through the Sec61p transport complex (Conesa et al., 2001). In the post-translational transport pathway, the nascent polypeptide is translated in the cytosol, and kept unfolded by interacting with Hsp70 chaperone and co-chaperones (Conesa et al., 2001). This complex is able to target ER through interaction with the membrane receptor Sec62p-Sec72p-Sec73p subcomplex (Conesa et al., 2001). The ER luminal chaperone binding immunoglobulin protein (BiP) and the membrane protein Sec63p assist the aforementioned complex to enter ER (Haßdenteufel et al., 2018).

**FIGURE 1:** Protein secretion pathway in filamentous fungi.

The second step is protein folding and modification in ER, which requires the assistance of a series of molecular chaperones and folding enzymes, including calnexin (ClxA), BiP, and protein disulfide isomerase (PDI) (Saloheimo and Pakula, 2012). For nascent peptides with correct folding, they are subjected to modifications such as glycosylation. As one of the most common and important post-translational modifications, glycosylation can significantly affect protein stability, localization, and secretion (Mitra et al., 2006). After proper folding and glycosylation, secreted proteins are transported extracellularly. On the other hand, the unfolded protein response (UPR) and ER-associated protein degradation (ERAD) are responsible for dealing with nascent peptides with incorrect folding (Bernasconi and Molinari, 2011; Wang et al., 2014). The UPR detects the presence of unfolded proteins in ER and induces the biosynthesis of chaperones and folding enzymes, while the ERAD degrades the misfolded proteins.

The third step is to transport the folded protein vesicles to the Golgi apparatus by fusion with target membrane, and secrete it to the extracellular environment (Spang, 2008). In filamentous fungi, Golgi-derived secretory vesicles are transmitted to the apical plasma membrane through apical vesicle clusters in Spitzenkörper (Virag and Harris, 2006). The formation, transportation and fusion of vesicles are mediated by a large number of proteins, including GTP-binding proteins (e.g., Sar, ARF) for vesicle budding, and Rab GTPases for fusion with Golgi (Hutagalung and Novick, 2011), etc. Specific fusion of vesicles with the target membrane is the critical process, which is mediated by soluble N-ethylmaleimide-sensitive factor-associated protein receptor (SNARE). Based on the localization, SNARE is divided into two categories: the vesicle SNARE (v-SNARE) and the target membrane SNARE (t-SNARE) (Söllner et al., 1993). In filamentous fungi, v-SNARE protein SNC1, and t-SNARE proteins SSO1 and SSO2, are involved in bubble fusion (Valkonen et al., 2007).

## Diverse Strategies for Enhanced Protein Expression and Secretion VIA Genetic Engineering

To enhance the protein expression and secretion in filamentous fungi, enhancing the intracellular protein production by optimization of the transcription and/or the codon of the target protein, is an effective strategy, as summarized in a few of reviews (Saunders et al., 1989; Jeenes et al., 1991; Nevalainen et al., 2005; Su et al., 2012). In order to bring new insights, we will discuss other genetic engineering strategies, including replacing original signal peptide with a more efficient one, fusion of heterologous protein to a naturally secreted one, regulation of UPR and ERAD, optimization of the intracellular transport process, construction of a protease-deficient strain, regulation of mycelium morphology, and optimization of the sterol regulatory element binding protein (SREBP) in this section (Table 1).

**TABLE 1:** Typical examples for genetic engineering of filamentous fungi for enhanced protein secretion.

**Protein of interest and its origin**	**Host**	**Strategy**	**Fold-change of protein secretion**	**References**
α-Galactosidase from *A. niger*	*A. niger*	Replacing the original signal peptide with a glucoamylase (GlaA) signal peptide in *A. niger*	Approximately 9-fold increase	Xu et al., 2018
Erythropoietin from human	*T. reesei*	Adopting the cellobiohydrolase I (CBH) signal peptide and optimizing *cbh1* promoter	Not applicable	Zhong et al., 2011
Chymosin from bovine	*A. oryzae*	Fusing target protein with a naturally secreted protein α-amylase	2-fold increase	Ohno et al., 2011
β-Glucuronidase from *A. niger*	*A. niger*	Regulating the UPR and ERAD by overexpression of *sttC* and deletion of *dorA*	Not quantified	Jacobs et al., 2009
Glucose oxidase from *A. niger*	*T. reesei*	Regulating the UPR and ERAD by overexpression of *bip1* or *hac1*	1.5–1.8-fold increase	Wu et al., 2017
Glucose oxidase from *T. reesei*	*T. reesei*	Optimizing the intracellular transport process by overexpression of *snc1*	2.2-fold increase	Wu et al., 2017
Prochymosin from bovine	*A. niger*	Optimizing the intracellular transport process by deletion of *Aovip36* or *Aoemp47*, and fusing the target protein with α-amylase	Approximately 2-fold increase	Hoang et al., 2015
Cellulase from *T. reesei*	*T. reesei*	Constructing a protease-deficient strain by deletion of *res-1*, *cre-1*, *gh1-1*, and *alp-1*	5-fold increase	Liu et al., 2017
Laccase from *Trametes versicolor*	*A. niger*	Constructing a protease-deficient strain by deletion of *pepAa*, *pepAb*, or *pepAd*	1.21–1.42-fold increase	Wang et al., 2008
Glucoamylase from *A. niger*	*A. niger*	Regulating mycelium morphology by deletion of *racA*	4-fold increase	Fiedler et al., 2018
Cellulase from *N. crassa*	*N. crassa*	Regulating SREBP by deletion of *dsc-2*, *tul-1*, *sah-2*, *dsc-4*, *scp-1*, or *rbd-2*	Not quantified	Reilly et al., 2015; Qin et al., 2017

## Replacing Original Signal Peptide With a More Efficient One

The signal peptide sequence plays vital role in protein secretion. Replacing with a more efficient peptide in target protein tends to increase its secretion efficiency. Xu et al. replaced the original signal peptide AglB of α-galactosidase with a glucoamylase (GlaA) signal peptide in *A. niger*, and the activity of extracellular α-galactosidase increased nearly ninefold (Xu et al., 2018). Wang et al. used green fluorescent protein as a reporter gene in *P. oxalicum* to test the secretion efficiency of three signal peptides, PoxGA15A, PoxAmy13A, and PoxCbhCel7A-2. Then they selected the optimal signal peptide PoxGA15A to drive the secretion of endogenous raw starch-degrading enzymes, which was 3.4 times higher than the parental strain (Wang et al., 2018).

## Fusion of Heterologous Protein to a Naturally Secreted One

Fusion of heterologous protein to a naturally secreted one can enhance protein stability, promote translocation, and prevent protein from degradation. The in-frame fusion of human protein granulocyte colony stimulating factor (G-CSF) with an endogenous highly secreted glucoamylase allowed secretion of 5–10 mg/L of G-CSF by *A. niger* (Kraševec et al., 2014). When bovine chymosin (CHY) was fused with alpha-amylase (AmyB), the engineered *A. oryzae* was able to produce two times higher amount of CHY than that with none fused CHY, while multiple genes involved in ER folding and protein secretion pathway increased significantly in the fused CHY producing strain (Ohno et al., 2011). It should be noted that the fusion carrier protein could greatly affect the secretion. In order to secrete *Escherichia coli* β-glucuronidase (GUS) protein in *Penicillium funiculosum*, researchers attempted to use xylanase as a carrier. The modular structure, a catalytic domain separated from the cellulose-binding domain by a linker with serine and threonine rich sequence, enables some xylanases as a group of unique protein carrier (Alcocer et al., 2003). It was reported that xylanase A (XYNA) is an effective carrier protein, while XYNB and XYNC are ineffective (Alcocer et al., 2003).

## Regulation of UPR and ERAD to Promote Protein Secretion

Correct protein folding is one of the many prerequisites to protein secretion. Abnormal folding proteins could form toxic aggregates exerting pressure on the ER, and trigger the feedback regulation called repression under secretion stress (RESS) to affect protein secretion (Pakula et al., 2003). UPR and ERAD are considered as two important ways to regulate protein folding, and enhanced protein secretion could be achieved via regulation of UPR and ERAD. For example, overexpression of the transcription factor *hac1* in *Aspergillus awamori* led to 7- and 2.8-fold increases in laccase and bovine prechymotrypsin production, respectively (Valkonen et al., 2003). Overexpression of *bip1* and *hac1* in *T. reesei* exhibited 1.5- and 1.8-fold improvement on secretion of an *A. niger* glucose oxidase (Wu et al., 2017).

To avoid degradation of some heterologous proteins or semi-folded proteins, deleting key genes involved in ERAD is a solution. Deletion of the ERAD factor *doaA* and overexpression of the oligosaccharyltransferase *sttC* responsible for glycosylation of secretory proteins (Yan and Lennarz, 2002) in *A. niger* caused an increase in β-glucuronidase yield (Jacobs et al., 2009). In addition, autophagy is considered as another way to degrade the misfolded proteins (Kario et al., 2011). Disruption of autophagy-related gene *aoatg15* in *A. oryzae* caused a threefold increase in secretion of bovine chymosin (Yoon et al., 2013).

Of particular note, manipulation of certain gene may cause quite different effects in different strains. For example, overexpression of *bip1* promoted protein secretion in *T. reesei* (Wu et al., 2017) and *A. awamori* (Lombraña et al., 2004), while reduced protein secretion was observed in *A. niger* by adopting the same strategy (Conesa et al., 2002). These effects could be attributed to the multifunction of BiP. BiP is able to promote protein translocation and folding, as well as to promote ER-associated protein degradation. Similarly, overexpression of *hac1* could promote protein secretion, which may also affect cell growth in certain strains (Valkonen et al., 2003; Carvalho et al., 2012). In addition, deletion of *derA* in *A. niger* can promote protein production (Carvalho et al., 2011), while deletion of the same gene affected the cell growth of *Aspergillus fumigatus* (Richie et al., 2011). It’s not difficult to see that the effect of protein secretion by regulating UPR and ERAD is host-dependent. Thus, a deep understanding of the complexity and specificity of the interactions between the components of the secretory pathway in a particular host is required prior to the manipulation.

## Optimization of the Intracellular Transport Process

Before being secreted outside, proteins are transported between ER and Golgi tendencies via vesicles. In this process, the ER-Golgi cargo receptor recruits the secreted proteins into the vesicles, thereby facilitating their transport (Dancourt and Barlowe, 2010). Optimization of the intracellular protein transport process allows enhanced protein secretion. In *A. oryzae*, the cargo receptor AoVip36 is localized in the ER and AoEmp47 is localized in the Golgi compartment. Deletion of AoVip36, responsible for anterograde transport, caused a 30% reduction of the endogenous α-amylase activity, and overexpression of this gene led to the increased secretion of EGFP (Hoang et al., 2015). In addition, deletion of *Aovip36* or *Aoemp47* increased the secretion of bovine prochymosin by approximately twofold (Hoang et al., 2015). In *Aspergillus nidulans*, gene *podB* is predicted to encode the subunit of the Golgi-conserved oligomeric complex (Gremillion et al., 2014), which is involved in Golgi retrograde vesicle transport, and affects cell polar growth, germination, and protein glycosylation (Wuestehube et al., 1996; Harris et al., 1999; Suvorova et al., 2002; Gremillion et al., 2014). A G-to-T mutation at nucleotide #751 in *podB1* led to significant increase in cellulase and xylanase activities (Boppidi et al., 2018). Wu et al. overexpressed *snc1* gene, which is involved in fusion of vesicles and plasma membrane, and observed a 2.2-fold increase in secretion of an *A. niger* glucose oxidase in *T. reesei* (Wu et al., 2017).

In addition to being successfully secreted outside, some heterologous proteins may be transported to the vacuole for degradation (Masai et al., 2003). Disruption of the vacuolar sorting receptor encoding gene *Aovps10* resulted in three and twofold increases in the production yields of bovine chymosin and human lysozyme in *A. oryzae*, respectively (Yoon et al., 2010).

## Construction of a Protease-Deficient Strain

The efficient production of certain endogenous protein in filamentous fungi disturbs the secretion of the protein of interest, and construction of a protease-deficient strain can strongly support the modification and secretion of the target protein. Disruption of alkaline serine protease SPW in *T. reesei* reduced the extracellular total protease activity by about 50%, and improved the production and stability of the heterologous alkaline endoglucanase EGV from *Humicola insolens* (Zhang et al., 2014). To construct a cellulase hyper-producing strain, β-glucosidase encoding gene *gh1-1*, alkaline protease encoding gene *alp-1*, and cellulase production related genes *cre-1* and *res-1* were simultaneously deleted in *Myceliophthora thermophile*. The secreted cellulase of the resulted strain was five times higher than that of the original strain (Liu et al., 2017).

## Regulation of Mycelium Morphology

Proteins are mainly secreted at vigorously growing mycelial tips in filamentous fungi (Wessels, 1993), and the mycelium morphology is especially important to protein secretion. The increased branching of the mycelium tip usually facilitates endogenous protein secretion. Lin et al. screened 90 morphological mutants of *Neurospora crassa* and found that disruption of *gul-1* led to a marked decrease in viscosity of the culture medium, while overexpression of *gul-1* led to a sharp increase in viscosity. In the *gul-1* disrupted strain, 25% and 56% increases were observed in the total extracellular protein concentration and β-glucosidase activity, respectively (Lin et al., 2018), suggesting that cell wall integrity has a significant effect on protein secretion. In *A. niger*, the Rho GTPase RacA regulates the polymerization and depolymerization of actin at the tip of mycelium (Kwon et al., 2011). When *racA* was deleted, the mycelial tip increased by about 20%, the number of secreted vesicles increased, and the secretion of glucoamylase increased 4 times as compared to the wild type strain (Fiedler et al., 2018). Similarly, deletion of *racA* resulted in a hyperbranched phenotype and three folds increase of cellulase activity in *T. reesei* (Fitz et al., 2019).

## Regulation of Srebp

In filamentous fungi, SREBP, responsible for regulating sterol homeostasis under challenging environments, is strongly associated with protein secretion, including linkages to the UPR (Qin et al., 2017) and formation of hyphae branches (Willger et al., 2008). After analysis the phenotype of a 567 single-gene deletion collection of *N. crassa*, researchers found that deletion of *dsc-2* and *tul-1 (dsc-1)* significantly increased the secretion of proteins (Reilly et al., 2015). In *Schizosaccharomyces pombe* and *A. fumigatus*, homologs of Dsc-2 and Tul-1 are part of the Golgi E3 ligase complex (Dsc complex), which can activate SREBP orthologs Sre1 and SreA through proteolytic cleavage (Lloyd et al., 2013). In addition, deletion of the unit of Dsc complex Dsc-4 and the Sre1/SreA homolog SAH-2 also showed a high secretion phenotype of cellulases (Reilly et al., 2015). Homologs of SAH-2 and TUL-1 from *N. crassa* are discovered in *T. reesei*, and their deletions enhanced the capability of protein secretion (Reilly et al., 2015). In a follow-up study, deletion of gene *scp-1* and *rbd-2*, encoding SREBP cleavage activating protein and rhomboid protease respectively, also led to the high producing phenotype of cellulose (Qin et al., 2017).

## Conclusion and Perspectives

Owing to the powerful protein secretion pathway, filamentous fungi are attractive cell factories for protein expression and secretion. For all the discussed strategies, replacing original signal peptide with a more efficient one, regulation of UPR and ERAD, optimization of the intracellular transport process, and construction of a protease-deficient strain have been successfully applied to improve the production of endogenous and heterologous proteins by filamentous fungi, while fusion of heterologous protein to a naturally secreted one is extremely effective for production of heterologous protein (Table 1). As for regulation of mycelium morphology and optimization of SREBP, although they were mainly adopted for production of endogenous protein, we believe that they are also applicable for production of heterologous protein. However, most efforts in genetic engineering of filamentous fungi for enhanced protein expression and secretion were solely based on the protein of interest, the secretory pathway or the host. Although these engineering strategies significantly improved target protein production, they were mainly related to single gene or pathway.

With the aid of multiple gene editing technologies (e.g., DNA recombination, RNAi, CRISPR-Cas), genome engineering strategies introduce deletion, insertion and/or point mutations across the genome via a trackable manner to accelerate strain evolution (Si et al., 2015). Compared with traditional metabolic engineering strategies, genome engineering allows rapid tracking and discovery of novel determinants (Xiao and Zhao, 2014; Si et al., 2017), editing of key determinant with single-nucleotide precision (Garst et al., 2017; Bao et al., 2018), or simultaneous manipulating multiple pathways (Barbieri et al., 2017; Liang et al., 2017). Apart from the unicellular model organisms (e.g., *Saccharomyces cerevisiae*), many filamentous fungi, particularly the mushroom-forming fungi, contain two different nuclei with different genetic contents (Gehrmann et al., 2018). In addition to the heterogeneity, many important medicinal mushrooms also exhibit low efficiency on gene transformation and homologous recombination (HR), which pose a great challenge to establish gene editing tools for genome engineering (Wang et al., 2020). To circumvent these difficulties, developing effective technologies for single spore isolation, gene delivery and/or improving HR efficiency are highly required in these filamentous fungi. It is notable that the target performances of the engineered strains, which are greatly improved by the aforementioned genome engineering strategies, can usually be screened out via cell growth or color. Thus, high-throughput screening methods are highly required to ensure the success of genome engineering. In fact, the fluorescence-activated cell sorting (FACS) assisted the intracellular protein production has been extensively adopted in filamentous fungi, but such strategy is difficult to screen out the beneficial mutants with enhanced protein secretion capacity (Throndset et al., 2010). To solve this problem, displaying the fluorescence protein on the cell surface, coupled by FACS, allows screening of the cellulose hypersecretors from *T. reesei* (Gao et al., 2018). As a promising alternative, the droplet-based microfluidic high-throughput screening platform has been established in *T. reesei* and *A. niger* (Beneyton et al., 2016; He et al., 2019). In future, we believe that harnessing the great potential of genome engineering will further increase protein expression and secretion by filamentous fungi.

## Author Contributions

CZ and HX designed this manuscript. QW and HX wrote this manuscript. QW, CZ, and HX revised this manuscript.

## Conflict of Interest

The authors declare that the research was conducted in the absence of any commercial or financial relationships that could be construed as a potential conflict of interest.

## Footnotes

1 https://amfep.org/about-enzymes/
